# Lesbian, gay, bisexual, and transgender (LGBT) health services in the United States: Origins, evolution, and contemporary landscape

**DOI:** 10.1371/journal.pone.0180544

**Published:** 2017-07-10

**Authors:** Alexander J. Martos, Patrick A. Wilson, Ilan H. Meyer

**Affiliations:** 1 Department of Sociomedical Sciences, Columbia University Mailman School of Public Health, New York, NY United States of America; 2 The Williams Institute, UCLA School of Law, Los Angeles, CA United States of America; University of New South Wales, AUSTRALIA

## Abstract

**Background:**

LGBT community organizations in the United States have been providing health services since at least the 1970s. However, available explanations for the origins of LGBT health services do not sufficiently explain why health in particular has been so closely and consistently linked to LGBT activism. Little is also known regarding how LGBT health services may have evolved over time with the growing scientific understanding of LGBT health needs.

**Methods:**

This study begins with a review of the early intersections of sexuality and health that led to an LGBT health movement in the United States, as well as the evolution of LGBT health services over time. Informed by this, an asset map displaying the location and types of services provided by “LGBT community health centers” today in relation to the population density of LGBT people was explored. An online search of LGBT community health centers was conducted between September–December, 2015. Organizational details, including physical addresses and the services provided, were confirmed via an online database of federally-registered non-profit organizations and organizational websites. The locations and types of services provided were analyzed and presented alongside county-level census data of same-sex households using geographic information system (GIS) software ArcGIS for Desktop.

**Findings:**

LGBT community health centers are concentrated within urban hubs and coastal states, and are more likely to be present in areas with a high density of same-sex couples. LGBT community health centers do not operate in 13 states. The most common health services provided are wellness programs, HIV/STI services, and counseling services.

**Conclusions:**

LGBT community health centers have adapted over time to meet the needs of LGBT people. However, significant gaps in service remain in the United States, and LGBT community health centers may require significant transformations going forward in order to continue serving LGBT people.

## Introduction

The LGBT health movement in the United States can be defined in terms of LGBT people providing for themselves a safe space for accessing healthcare services [1–6]. LGBT health services, or health services offered through LGBT community organizations, have been available since at least the 1970s [7]. Available explanations for the origins of LGBT health services, such as the increased community mobilization and explicit rejection of homophobia following the Stonewall Riots of 1969 [5], do not sufficiently explain why health in particular has been so closely and consistently linked to LGBT activism. Little is also known regarding how LGBT health services may have evolved over time with the growing scientific understanding of LGBT health needs. LGBT community organizations provided health services to at least 300,000 clients in 2015 [8], suggesting that they still constitute a significant proportion of the healthcare landscape for LGBT people today.

Researchers have sought to understand LGBT patients’ experiences accessing healthcare services and preferences for care [9–14]. These studies focus predominantly on the general population healthcare landscape and offer limited consideration for LGBT health services. This study is an effort to understand the origins of the LGBT health movement and to characterize the landscape of LGBT health services today in the United States. We begin with a review of early intersections of sexuality and health and the evolution of LGBT health services over time. Informed by this, we present an asset map displaying the location and types of services provided by LGBT community health centers today in relation to the population density of LGBT people.

Given the diversity of the LGBT community, it is prudent to describe how identity labels are utilized in describing the findings below. For example, although not everyone outside of heterosexual, cisgender (i.e., people whose sex assigned at birth is consistent with their gender identity) identities would describe themselves as lesbian, gay, bisexual, or transgender, the term LGBT is used to collectively refer all sexual minority, transgender, or gender non-conforming people. Other terms will be incorporated to describe particular political, medical, or social moments or perspectives, rather than LGBT people themselves. For example, the term “homosexual” was used early in medical literature to refer to those with same-sex attraction, and was often extended to those who may today identify today as bisexual or transgender as a result of the limited terminology used at the time. The term “homophile movement” was subsequently adopted by many LGBT people who began organizing themselves in the 1950s. For a more in-depth overview of how these community identity labels have changed over time, both socially and scientifically, see Armstrong (2002), D’Emilio (2012), Weststrate & McLean (2010), and Young & Meyer (2005) [15–18]. Finally, LGB and LGBT are used differentially to accurately describe the inclusion or exclusion of transgender (and other gender non-conforming people) from the LGBT health movement.

## Origins of LGBT (health) movements and services

Michel Foucault’s *The History of Sexuality* [19] explores how notions of sexuality have been constructed, and how the boundaries of “legitimate” sexuality have been contested, historically. There is no clear beginning to the relationships between sexuality, social and political movements, and health. But the interplay of these factors in the formation of LGBT identities in the United States has origins in the mid-20^th^ Century [16]. Prior to adopting more consolidated identities of lesbian, gay, bisexual, and transgender, unorganized and isolated individuals first sought to identify and connect with each other in the politically and socially hostile climate following World War II [20]. In the midst of 1950s McCarthyism, two organizations formed that would greatly influence the trajectory of what would ultimately become “LGBT” people in the United States: The Mattachine Society [20] and the Daughters of Bilitis [21]. Both groups organized in secrecy, regularly published and distributed magazines and newsletters to subscribing members that debated the meaning of homosexuality, and provided medical professionals’ perspectives on homosexuality [16, 20, 21]. Both groups came to promote the notion that sexuality was constitutional to one’s identity, and that subscribing members were a discriminated minority [20]. These moves toward self-acceptance and identity development would ultimately encourage public advocacy for the rights and social acceptance of a broader community.

Concurrent with this early mobilization were several other pivotal developments that helped the increasingly organized groups of LGBT people challenge the illness model of homosexuality. Several studies helped make a case for same-sex sexual behaviors as a normal and acceptable form of sexual expression, including Alfred Kinsey’s studies demonstrating the high frequency of same-sex behaviors among men [22] and women [23], Ford and Beach’s (1951) reports that same-sex sexual behaviors occurred naturally both within various animal species around the world and across numerous cultures globally [24], and Evelyn Hooker’s (1957) study found no mental health differences between heterosexual and homosexual men other than their status as homosexuals [25]. Early forms of activism among LGBT people leveraged these studies in order to dismantle the definition of homosexuality as a psychological disorder.

In 1960, the first transgender-specific magazine in the United States, *Transvestia*, was published [26]. Like the publications distributed by the Mattachine Society and Daughters of Bilitis, *Transvestia* incorporated social commentary, educational outreach, and readers’ own autobiographical submissions. It also argued against the criminalization of gender non-conforming dress and promoted early ideas of transgender people as a minority community [26]. Transgender people continued to organize throughout the 1960s, developing community and activist organizations and promoting research into medical gender confirmation procedures [26, 27].

These efforts were vital in pushing back against anti-homosexual political action that prevailed following 1950s McCarthyism. The rise of consumerism, a growing working class of women, and feminist and civil rights critiques following World War II resulted in many sexual and gender norms being dissolved or reconfigured. In response to the growing challenges to sexual and gender norms, federal, state, and local governments mobilized their resources “against the underground sexual world” ([28], pp. 288), framing “homosexuals” as both the source of social decay and a threat to national security. LGBT people were sought out, arrested, and exposed under the guise of protecting the social order.

In such a hostile climate, new forms of political and social organizing and advocacy were needed [28]. The Stonewall riots of 1969 represent a significant turning point for LGBT people, who not only protested against the frequent police raids in New York City but also organized a nationwide, grassroots liberation movement [16]. Though not by any means the first form of public protest from LGBT people [29], it served as a very visible and forceful catalyst to national organizing as sexual minorities began identifying services they could not adequately receive elsewhere and providing for themselves [5, 16].

Over 1,000 community-based organizations serving LGBT people emerged in the 1970s [16], following the opening of the first LGBT community center in Los Angeles in 1969 [7]. However, upon the removal of homosexuality from the American Psychiatric Association’s Diagnostic and Statistical Manual (DSM) in 1973 [30], a noticeable break occurred between transgender people and lesbians, gay men, and bisexuals (LGBs). Transgender people, once a part of the collectives advocating for a progressive shift in how sexuality was viewed socially and politically, were entered into the DSM under a new pathology, “Gender Identity Disorder of Childhood” [31]. Transgender people were then systematically excluded from LGB groups, who wanted to distance themselves from notions of deviance and medical pathology that transgender people now carried the burden of [32]. Likewise, feminist groups resisted the inclusion of transgender people, leaving them with few social and political allies throughout the 1970s and 1980s [26]. Medical, legal, and psychotherapeutic professionals working with transgender people continued to provide healthcare, conduct research, and develop standards of care via professional organizations like the World Professional Association for Transgender Health (WPATH; formerly the Harry Benjamin International Gender Dysphoria Association, founded in 1966) [26, 33]. Such organizations were among the few resources that remained to transgender people through the 1980s.

With homosexuality no longer included in the DSM, large numbers of LGB people were able to create visible communities in urban hubs [4]. Though these communities by no means flourished in all areas, the rapid growth of LGB organizations throughout the country enabled the once disparate people to share information across communities and better serve their local needs. It was soon recognized that many LGB people were stigmatized when accessing services in general healthcare settings, and as a result many LGB organizations took it upon themselves to offer an alternative source of care [3, 6, 34].

## Evolution of LGB(T) health movement and services

The infrastructure for community-based health services was being established with the proliferation of LGB community centers throughout the country. However, lessons learned within the women’s health movement introduced the idea of uniquely “LGB” health issues. In 1973, the Boston Women’s Health Book Collective published the second edition of *Our Bodies*, *Ourselves* [35, 36]. As a part of recognizing women’s unique healthcare needs, one chapter focused specifically on lesbian health issues and the shortcomings of medicine and healthcare in meeting their needs. LGB community centers and activists began to consider the possibility of unique health issues and disparities in need of specialized attention.

These programmatic shifts are visible within both emerging and pre-established community centers of the 1970s. Fenway Community Health, founded in 1971 in Boston, Massachusetts, was not initially established as an LGB community health center, but became the first community health center to develop expertise in LGB health services in response to the demographic needs of its own staff and clients [37]. A similar expansion of services into health occurred in Los Angeles, New York, Chicago, and Philadelphia [5, 38]. By the mid-1980s, the National Gay Task Force listed over 100 clinics and medical service programs and over 300 counseling and mental health programs, with services ranging from testing and treatment for sexually transmitted infection to counseling and care for substance users, that were openly LGBT friendly and accepting [5].

This combined community and institutional organizing would prove invaluable by the onset of HIV/AIDS in the 1980s. The federal government, and particularly President Regan, were slow to respond to the epidemic [2], but the HIV/AIDS crisis raised the stakes for LGB people to gain access to additional health resources. Many LGB organizations and activists leveraged the health implications of HIV/AIDS to raise awareness about such issues as domestic partnerships, access to the sick and dying, inheritance, and housing [29]. At the community level, gay men and their allies–particularly lesbians drawing upon their experiences in the reproductive rights and women’s movements–organized themselves into activist and advocacy groups such as the Gay Men’s Health Crisis in 1982 [39], and ACT UP in 1987 [2]. Meetings held by these groups disseminated the latest HIV research and prevention strategies, developed (often radical and militant) strategies for social and political advocacy, and identified and organized social and healthcare services for men with HIV and AIDS who were unable to receive adequate services elsewhere [2, 3]. LGB organizations rapidly responded by offering emotional and practical support to those affected by HIV, counseling, sex education, home-based hospice care, housing and other social services [1, 2].

The action taken at the community level resulted in increased public awareness of HIV and AIDS and initiated action at the federal level. LGB health professionals and activists took advantage of the growing public attention by applying pressure to federal agencies and professional organizations such as the National Institute of Health (NIH), the Food and Drug Administration (FDA), the Centers for Disease Control and Prevention (CDC), the American Public Health Association (APHA), and the American Medical Association (AMA) [3, 40]. Their goals were to raise national awareness about HIV/AIDS and the crisis among gay men, accelerate the clinical trial process for new treatments, and allocate additional research focus to gay men in particular [2, 3].

However, the narrow focus on HIV over the course of the 1980s and 1990s re-associated homosexuality with illness after long-fought struggles to disassociate from the medical field [41, 42]. Though large amounts of federal funding were made available to research HIV among gay men, little attention was given to other health issues among either gay men or LGBs in general [3]. In an effort to ensure that HIV would not dominate the discourse around LGB health issues, “a small and pioneering group of academic researchers began seeking to fill the vacuum of knowledge about lesbian and gay, and particularly lesbian, health concerns” ([3], pp. 138). At the same time, transgender people re-emerged to advocate for their own uniquely transgender health issues, including issues related to HIV and gender confirmation [43, 44].

Little has been written on the political, social, and historical milestones for transgender people during the 1980s. Transgender communities are believed to have concentrated “more on providing mutual aid and support to their members than on broader social activism” during this time ([26], pp.113). On the other hand, the 1990s saw a burst of activity that sparked an increase in activism. Ongoing debates within feminist studies and theory resulted in the development of a queer theory that legitimized transgender identities. HIV research also began to recognize transgender people as a “vulnerable” population in the era of AIDS, and transgender people were increasingly incorporated into human rights laws and protections within municipalities throughout the United States [26]. Once again advocating for issues as a collective, LGBT people together produced a large body of research pointing to diverse and complex health disparities [45–49]. Formerly LGB organizations began re-branding themselves as inclusive of transgender individuals, and a focus on LGBT health took shape at both community and national levels [3].

The collective efforts of LGBT community centers, activists, and professionals culminated in a variety of events that aided LGBT people in gaining national recognition as an underserved population in health. These include: professional health associations’ recognition of LGBT caucuses [5]; the 1999 report on lesbian health by the Institute of Medicine (IOM) [50]; a white paper sponsored by the Gay and Lesbian Medical Association (GLMA) leading to the inclusion of LGB people in Healthy People 2010 [51]; the first special issue on LGBT health by the American Journal of Public Health (AJPH) in 2001 [52]; the 2002 recognition of the first LGBT community health center as a Federally-Qualified Health Center (FQHC) by the Health Resources and Services Administration (HRSA) Bureau of Primary Health Care [53, 54], ensuring federal funding and reimbursement for health services provided by LGBT health clinics; and finally the inclusion of LGBT people collectively within Healthy People 2020 [55]. In 2011, the IOM published a comprehensive report on LGBT health entitled “The health of lesbian, gay, bisexual, and transgender people: Building a foundation for better understanding” [56]. In it, they synthesized decades of research on LGBT health in order to summarize what was known about the disproportionate burden of disease among LGBT people and areas for future research.

Health issues recognized by the IOM report as pertinent to either all or particular subgroups of LGBT people include: Anxiety; access and other barriers to quality care; depression; suicide and suicidal ideation; eating disorders; adolescent pregnancy; obesity; HIV and other sexually transmitted infections; breast cancer; anal cancer; cervical cancer; bullying and harassment; erectile dysfunction; substance abuse (including cigarettes, alcohol, and other drugs); cardiovascular disease; and elevated rates of other cancers possibly associated with hormone treatments for transgender individuals [57]. Each of these can be recognized as relevant health concerns for LGBT populations, but researchers and community members have questioned how disproportionate health burdens could or should translate to concrete health service [5, 57]. Although no clear consensus has been reached, LGBT community health centers have developed LGBT health services that address the physical health, mental health, social, and educational needs of the LGBT people.

Guided by this review of the literature, we now turn to assess the scope of LGBT health services in the United States today. Publicly available data were analyzed and used to generate a United States LGBT community health center asset map. We then discuss how the LGBT health movement has shaped the contemporary landscape of LGBT health services, current gaps in service, and consider how social and political changes may influence the LGBT health service landscape moving forward.

## Contemporary landscape of LGBT health services

### Methods

#### Definitions and criteria

To generate an asset map of the contemporary landscape of LGBT health services, several key constructs required operationalization. Based upon findings from the literature review, definitions and criteria for LGBT community centers and LGBT community health centers were generated. These definitions and criteria ensured that all organizations and service sites identified during data collection were appropriately categorized and, if necessary, excluded from analyses. Definitions and criteria are included in Table 1. FQHCs are also included in Table 1 in order to contrast our own definition of and criteria for LGBT community health centers with the stringent criteria that must be met in order to be recognized federally as a community health center. Although FQHCs are able to provide much more comprehensive care than the LGBT community health centers we define here, many LGBT community health centers operate in smaller capacities and provide a variety of health services to their local community members. For example, while only 14 of the more than 1,100 federally-funded Community Health Centers focus on LGBT populations [58–60], CenterLink, a coalition of 180 LGBT community organizations, identified at least 62 LGBT organizations providing health services [7]. CenterLink publishes a biennual report on the status and service efforts of LGBT community organizations throughout the United States.

**Table 1:** Center types, definitions, and criteria for data collection.

	Definition	Criteria	Operationalization
LGBT Community Center	Federally registered 501(c)(3) non-profit organizations that operate within a physical space where services are provided explicitly (within the organizational mission statement) for lesbian, gay, bisexual, and/or transgender people. As such, these organizations cater to the needs of LGBT people within a specified geographic area who can access the services provided.	- Explicitly serves lesbian, gay, bisexual, and/or transgender populations.	- Mission statement identifies lesbian, gay, bisexual, and/or transgender populations as intended recipients of services.
		- Registered non-profit organization with Internal Revenue Services (IRS).	- 2014 registration with IRS confirmed via guidestar, or that of a fiscally supporting organization.
		- Has a physical space where services are offered.	- Organization identifies (online, via IRS registation or telephone) a physical address where repeated services are offered at least once monthly.
		- Currently in operation.	- 2014 registration with IRS confirmed via guidestar, or that of a fiscally supporting organization.
		- Operates at local, state, or regional levels (i.e., not national).	- Mission statement specifies a non-national service area.
LGBT Community Health Center	An LGBT community center that regularly provides at least one health service in-house.	- LGBT community center	- Meets criteria for LGBT community center displayed above.
		- Health Services	- At least one LGBT health service, as identified by CenterLink's 2014 community center survey (general medical services; pharmacy services; STD/HIV services; counseling; peer support groups; 12-step programs; psychiatric services; anti-violence programming; wellness programs), is offered within the physical space operated by the organization at least one monthly.
Federally-Qualified Health Center (FQHC)	Outpatient clinics that qualify for specific reimbursement systems under Medicare and Medicaid (RAC, 2015).	- Offer services to all persons, regardless of the person's ability to pay.	Applications to be recognized as an FQHC are received and reviewed by the Health Resources and Services Administration Bureau of Primary Health Care.
		- Establish a sliding fee discount program.	
		- Be a nonprofit or public organization.	
		- Be community-based, with the majority of their coverning board of directors composed of their patients.	
		- Serve a medically underserved area or population. In this case, the medically underserved population would be defined as a lesbian, gay, bisexual, and/or transgender population.	
		- Provide comprehensive primary care services.	
		- Have an ongoing quality assurance program.	

#### Data collection

In 2014, CenterLink contacted 211 (member and non-member) LGBT community organizations within the United States and Puerto Rico. Of those, 111 responded to the agency’s online survey, representing 32 states, Washington, D.C., and Puerto Rico. Responding organizations were predominantly independent entities, however, a few (13%) were affiliates of other organizations (e.g. local community health groups). Most organizations occupied a physical space, but 6% operated solely through phone or mobile van services only [7].

Initial records for LGBT organizations and their respective service sites were created using the lists of 180 CenterLink member organizations and 111 respondents to their 2014 biannual LGBT community center survey [7, 61]. These lists were not mutually exclusive, and not all respondents to the biannual survey were CenterLink members, resulting in an initial list of 193 organizations and service sites. We then searched public records for each organization using GuideStar, a database of IRS-registered non-profit organizations, to confirm non-profit status. Any new organizations that was identified via the GuideStar search were added to the list. Additional organizations were also identified using the “Resources” (or similar topic) section of organizational websites. In the event that any of the criteria for LGBT community health centers was unavailable on an organizational website, organizations were contacted by telephone to confirm the missing data. Organizations that did not meet the criteria for LGBT community centers, or for which the criteria could not be confirmed via online search or telephone call, were excluded. Data collection occurred between September–December, 2015. In June, 2016, CenterLink published their 2016 LGBT Community Center Survey Report [8]. Ten new organizations were included that had not been otherwise identified, of which two met the criteria for an LGBT community center. Neither met the criteria for an LGBT community health center.

LGBT health services were categorized according to CenterLink & Movement Advancement Project’s (MAP’s) 2014 findings [7]. These include: general medical services; pharmacy services; STD/HIV services (i.e. prevention, testing, treatment, counseling, etc.); individual, group, couples, and family counseling; peer support groups; 12-step programs; psychiatric services; anti-violence programming; and wellness programs and services (e.g. healthy eating, active living, cancer support, and other healthy living programs and support groups). Additional categories were created for organizations whose health services did not fit within the above categories. These include: transgender care (specialized physical and mental health services for transgender patients), addiction services (syringe exchange and recovery programs), and health insurance enrollment programs. LGBT community centers that operated a physical health clinic were also identified, and were defined as clinical spaces operated by trained and licensed healthcare personnel. These include but are not limited to primary care clinics in that health clinics may specialize in specific services (e.g., testing and treatment of sexually transmitted infections) rather than offer the full service scope of primary care. Community health centers that offer health services in the absence of a trained and licensed professional (e.g., cancer support groups, HIV prevention programs, 12-step programs) would not be qualify as operating clinical spaces.

In all, 435 records were created during the search for LGBT community health centers. Of these 435 records, 129 (29.7%) did not meet the criteria to be defined as an LGBT community center (Fig 1). The remaining 306 LGBT community center service sites were operated by 219 independent LGBT community centers. Of those, 213 (69.6%) were identified as LGBT community health center service sites, which were operated by 147 independent LGBT community health centers.

**Fig 1:** Identification of LGBT community health centers.

#### Data analysis

Data previously compiled by the Williams Institute [62] in which census data was used to describe same-sex households per county in the United States [63] were uploaded into Geographic Information System (GIS) ArcGIS Desktop software. Same-sex households, identified using 2010 census data, is used in this study as a proxy for local LGBT population density. Using the GIS software, same-sex household data was joined to a Tiger/Line shapefile representing the geographic boundaries of United States counties. Doing so associated United States counties within the electronic map shapefile with their relative number of same-sex households. The county shapefile was then overlaid above a United States shapefile displaying the state and national boundaries of the United States. Next, county areas were filled by graduated colors representing the relative proportion of same-sex households to all households per county. These groups were defined according to the Esri version of Jenks natural breaks classification, which “creates grouped classes according to clusters and gaps in the data” [64, p. 134]. Finally, LGBT community health centers were geocoded, or linked to a specific geographic location within the United States map, in order to display their location relative to the local same-sex population density. A 60-mile buffer was created around each LGBT community health center to represent the geographic coverage area for each center. The 60 miles radius was chosen to approximate a one-hour drive from each center.

Centroid locations, or the most central point of each county polygon, were calculated using ArcGIS in order to determine approximate distances between each county center and its nearest LGBT community health center. The dataset was then exported to STATA 12.1 containing the number of same-sex households by county and the distance from county center to the nearest LGBT community health center. Linear regression was run to determine whether the local LGBT population density was significantly associated with the distance to the nearest LGBT community health center.

### Results

Fig 2 displays the locations of all 213 LGBT community health centers in relation to LGBT population density by county. Clusters of LGBT community health centers are located on both coasts of the continental United States, with fewer or no health centers located in the center, Alaska, or Hawaii. Within the continental United States, no LGBT community health centers were identified in Arkansas, Iowa, Kansas, Louisiana, Maine, Nebraska, New Hampshire, North Dakota, South Dakota, West Virginia, and Wyoming. As seen, LGBT community centers are closely aligned with same-sex household population density (this association is statistically significant as tested by a bivariate linear regression predicting the locations of LGBT community health centers from the number of same-sex households by county, β = -0.00049, S.E. = 0.00015, p = 0.001).

**Fig 2:** 60-mile radius surrounding all LGBT community health centers.

Figs 3 and 4 display the locations of LGBT community health centers that operate general health clinics (Fig 3) and those whose health clinics offer transgender care services specifically (Fig 4). Fig 3 shows that restricting to health clinic only narrows the number of locales to just 61 LGBT community health centers in only 11 states (Alabama, California, Connecticut, Florida, Georgia, Pennsylvania, Illinois, Massachusetts, Maryland, New York, Texas) and the District of Columbia. Fig 4 displays community health centers offering transgender services, specifically, which further reduced the number of centers to only 21, which are available in only 9 states (California, Connecticut, Florida, Georgia, Pennsylvania, Illinois, Massachusetts, New York, Texas) and the District of Columbia. Both general health clinics and health clinics that specialize in transgender health are concentrated in the northeastern United States.

**Fig 3:** 60-mile radius surrounding LGBT community health centers operating a health clinic.

**Fig 4:** 60-mile radius surrounding LGBT community health centers offering transgender care.

Fig 5 displays the type of services provided across all LGBT community health centers. Most health centers provide wellness programs and services (n = 153; 72%), HIV/STI services (n = 138; 65%), and counseling services (n = 110; 52%), with psychiatric (n = 7; 3%) and pharmacy (n = 16; 8%) services being the least available across all health centers.

**Fig 5:** Health services provided by LGBT community health centers.

## Discussion

The history of the LGBT health movement in the United States is inextricably linked to long-running political, social, and scientific associations between LGBT people and health. Consistent with Foucault’s understanding of the relationship between sexuality and power, efforts to gain social and legal recognition as a minority group required LGBT people to also challenge notions of “normal” and “healthy” sexuality [19]. Early efforts to protect LGBT people against societal stigma and prejudice motivated LGBT communities to provide themselves with better health services than they could not obtain in general population settings. In their earliest form these health services consisted predominantly of general medical, mental health, and sexual health services at LGBT organizations operating small health clinics [5, 37, 38]. These organizations soon included such specialized services as hospice, grief counseling, cancer prevention, peer support groups, and 12-step programs in the era of HIV, the stigma from which left many without access to care in the general population healthcare settings [1, 2].

LGBT health services have continued to evolve and expand in accordance with social change and medical advances. For example, hospice care services have presumably diminished within LGBT community health centers as HIV-related morbidity and mortality decreased, while counseling services remain common and have expanded in the types of counseling services available. The expansion of services over time demonstrates that, whether offering highly technical and specialized medical care or preventative and wellness services, a majority of LGBT community organizations have made health a priority. The high prevalence of wellness services suggests that even organizations with limited resources may be able to engage with health promotion and prevention efforts in their communities.

This study highlights a number of challenges with regard to accessing LGBT health services. First, as Fig 2 demonstrates, while significant proportions of LGBT people living on either coast live within 60-miles of an LGBT community health center, the central states are largely under-served. Thirteen states are devoid of LGBT community health centers altogether. And while we used a 60-mile radius as an indicator of proximity, even a 60-mile radius may not represent accessibility in the dense urban and coastal hubs. Moreover, proximity to any one LGBT community health center does not necessarily mean access to comprehensive LGBT health services given that each LGBT community health center provides a different combination of health services.

At the same time, we should not assume that a lack of LGBT community health centers equates to a lack of culturally competent health services. There are alternative venues where LGBT people could access health services, such as women’s clinics or private practices, that may provide quality care to them. Similarly, although LGBT community health centers may be more aware of and sensitive to the needs of clients with diverse gender and sexual identities than general healthcare providers, this capacity for greater cultural competence does not necessarily extend across racial/ethnic groups, socioeconomic diversity, and immigration status. Black LGBT people, for example may still feel a lack of competency from, or a level of discomfort with, LGBT-specific providers who are not Black themselves [10].

The purpose of this study is not to definitively determine all the places LGBT people can and do access culturally competent care. With that said, our own findings suggest that CenterLink and MAP have likely greatly under-reported the number of LGBT people served in 2015, as their estimate of 300,000 people served is based upon data reported by only 62 organizations [8]. LGBT community health centers continue to be a valuable resource to LGBT people, and how these resources are invested in going forward is a matter of great concern.

### Limitations

The research conducted as a part of this study is limited in a few ways. First, we cannot claim to represent all LGBT community health centers. Although we had criteria for defining and categorized organizations during data collection, there was nonetheless room for error. Information available online was assumed to be accurate, particularly including information regarding the services provided. However, if an organization had recently added or removed services without updating the website than their classification as an LGBT health center (or not) may be inaccurate. Also, our findings represent an overall snapshot of the LGBT community health centers and services provided between September–December of 2015. The nature of studying or working with community-based organizations requires some allowances for imperfections in the data collected. One consequence of being a small, new, or under-resourced LGBT community health center–as many of the organizations included in our study are [8]–is that the services they provide may change over time or even cease to exist. This may be the result of organizations merging together, shifting the services provided according to the demands, the availability of new funding opportunities, the withdrawal of funding, and changes in personnel. Finally, our findings only describe the availability of services offered by LGBT community health centers, not on the quality of services or even the extent to which any services are utilized. Our goal here was to discuss the broader scope of what LGBT health services look like today, and we believe we have achieved that goal.

This study is also limited in its ability to speak to the wide diversity of LGBT experiences. For example, the literature review contains several significant gaps with respect to the unique roles and experiences of LGBT racial/ethnic minorities, bisexuals, and transgender people within the LGBT health movement. Although people whose identities lie within each of these categories undoubtedly played important roles in the broader “LGBT” movement, their stories may often be subsumed under, or even appropriated by, the largely White, middle-class, gay narratives dominating the literature [32, 65]. The present study cannot speak to the involvement of these populations in the LGBT health movement in the absence of literature on the subject. Similarly, without assessments of the origins, evolution, and contemporary landscape of LGBT health movements internationally, it is not possible to situate these findings within the broader story of LGBT people globally. We hope that our research encourages future studies to explore the wide diversity of LGBT people and their experiences within health movements in different regions of the world and over time.

Finally, the census data representing LGBT population density do not adequately represent the actual size of local LGBT populations or its diversity. One reason being that not all LGBT people have or live with their partners, and another being that not all would feel comfortable identifying themselves as living in a same-sex household. But this approach also fails to capture bisexual and transgender people in opposite-sex households. These numerous limitations to determining the geographic distribution of LGBT people, and particularly bisexual and transgender people, in turn limit the study’s ability to fully assess the distribution of LGBT health services. For example, it may be that bisexual and transgender people are more highly concentrated in distinct areas from lesbians and gay men, but that those communities are not visible within the census data. In spite of these limitations, this approach using census data remains a useful metric for determining where LGBT people may be more highly concentrated. With no national census data on sexual orientation of individuals, this is the most comprehensive national data currently available for estimating the geographic distribution of the LGBT people.

### Conclusion

As acceptance of LGBT people increases [66, 67], the need for specialized services may decrease. However, it remains unclear what the path forward will be for LGBT community health centers. It is possible that there will always be a need for LGBT-specific health services no matter what the level of social acceptance becomes. In this case, we may see continuation of the increase in the numbers of LGBT health centers, their spread into parts of the country where they are now absent, and greater sophistication of their services regarding the needs of diverse subgroups of the LGBT population (e.g. young Black gay men, older Latina lesbians).

But it is also possible that we will see a reduction or consolidation of LGBT health services as LGBT people find comparable services at general, not LGBT-specific, clinics. Koester and colleagues [9] explored this among gay and bisexual men, concluding that gay and bisexual men may come to prefer having both LGBT-specific and general population healthcare services available to them, but would utilize particular kinds of services in each setting. For example, young, HIV-negative gay and bisexual men reported a preference for separating sexual health services, which they sought in LGBT-specific centers, and other general health services, which they sought in general population settings. In this case of segmented care, LGBT community health centers would need to grow their understanding of LGBT peoples’ healthcare preferences in order to provide highly tailored services when comprehensive care is not an organizational option.

LGBT people may also eventually choose healthcare settings where all their healthcare needs can be consolidated. Differences in sexual orientation disclosure rates to healthcare providers between rural and urban settings suggests that LGBT people may feel more comfortable with general population healthcare providers in urban settings [68]. A shift away from LGBT community health centers may then begin in urban centers, where there is greater acceptance of LGBT people, and would suggest a greater need for LGBT organizations to re-direct services toward rural areas, where LGBT people are more likely to be shunned, or for services, support and consultation to be made available online or via telephone in order to accommodate the needs of those outside of urban centers. Also, to the extent that younger people would become less likely to identify LGBT labels [69, 70], traditional LGBT organizations may struggle to appeal to future generations. Future studies on LGBT healthcare should consider preferences for venue, provider, and services, as well as overall satisfaction, access and utilization across LGBT sub-populations (e.g., race/ethnicity, gender identity, age cohort) and geographic region.

Additionally, preferences for consolidated services may lead LGBT community health centers to much more closely resemble (or ultimately gain recognition as) FQHCs in order to provide consolidated care and attract a greater client base. This may be particularly true in rural settings, as FQHCs have demonstrated a history of providing quality care to socially and medically disadvantaged patients [71, 72]. LGBT community health centers have increasingly been recognized as FQHCs over the past 15 years, through a number of dramatic shifts in political, social, and health care system landscapes. Although it is difficult to assess how, for example, the implementation of the Affordable Care Act (United States healthcare legislation passed in 2010 that increased access to health insurance for citizens beginning in 2014) influenced the LGBT health service landscape during the period of data collection for the present study, it is notable that LGBT community health centers began gaining recognition as FQHCs long before, and throughout, its implementation. Furthermore, with only 14 of the LGBT community health centers recognized as FQHCs, and their long history in the United States, it is safe to assume that they will remain prominent in the LGBT healthcare landscape for many years to come.

The LGBT health movement has generated over 200 LGBT community health centers providing services to LGBT people throughout the United States. Although many states and communities remain un- or under-served, it is clear that the LGBT health movement has grown greatly since its earliest manifestations in the 1950s to serve the health needs of LGBT people in the United States. With many social and political changes in the U.S., the long-term future of LGBT health services is uncertain. It is vital that researchers explore the forces that shape health care provision for LGBT people and how the immensely diverse populations of LGBT people will choose to access these services. The LGBT health movement has a complex task of working toward the dual goals of better tailoring LGBT health services to the needs of LGBT people as well as ensuring that they all have access to health services within safe spaces.

## Supporting information

S1 File LGBT community center data, geocoded. (XLSX)

S2 File Number of same-sex couples by United States county, United States census. (XLSX)
